The article "Deep Learning for Intelligent Recognition and Prediction of Endometrial Cancer" was published in 2021. Journal: J Healthc Eng.

# Deep Learning for Intelligent Recognition and Prediction of Endometrial Cancer

**DOI:** 10.1155/2021/1148309

**Published:** 2021-08-26

**Authors:** Yan Zhang, Cuilan Gong, Ling Zheng, Xiaoyan Li, Xiaomei Yang

**Affiliations:** ^1^Department of Obstetrics, Huangdao District Hospital of Traditional Chinese Medicine, Qingdao 266500, China; ^2^Department of Gynaecology, Huangdao District Chinese Medicine Hospital, Qingdao 266500, China

## Abstract

The aim of the study was to investigate the intelligent recognition of radiomics based on the convolutional neural network (CNN) in predicting endometrial cancer (EC). In this study, 158 patients with EC in hospital were selected as the research objects and divided into a training group and a test group. All the patients underwent magnetic resonance imaging (MRI) before surgery. Based on the CNN, the imaging model of EC prediction was constructed according to the characteristics. Besides, the comprehensive prediction model was established through the clinical information and imaging parameters. The results showed that the area under the working characteristic curve (AUC) of the radiomics model and comprehensive prediction model was 0.897 and 0.913 in the training group, respectively. In addition, the AUC of the radiomics model was 0.889 in the test group and that of the comprehensive prediction model was 0.897. The comprehensive prediction model was established through specific imaging parameters and clinical pathological information, and its prediction performance was good, indicating that radiomics parameters could be applied as noninvasive markers to predict EC.

## 1. Introduction

EC is a group of epithelial malignant tumors that occur in the endometrium, the most frequent is adenocarcinoma originating from the endometrial glands [1]. What is more, EC often emerges in postmenopausal and perimenopausal women. It is one of the most common tumors of the female reproductive system, with nearly 200,000 new cases every year [2]. Among the gynecological malignant tumors that cause death, it ranks third after ovarian cancer and cervical cancer. With the rapid development of social economy, the incidence of EC is gradually increasing in China, and it is the second place among malignant tumors [3]. At present, the cause of EC is still unclear. Some scholars have pointed out that its risk factors are related to fertility, hormones, metabolism, and physiological behavior [4]. Endometrial hyperplasia is the pathological change of the endometrium before canceration and has the potential to deteriorate. The morphology of atypical endometrial hyperplasia is similar to that of EC, and it is difficult to distinguish in clinical diagnosis [5]. Based on the danger of endometrial hyperplasia and the difficulty of clinical diagnosis, it is necessary to find a method that can intelligently identify normal endometrial, endometrial hyperplasia, and endometrial cancerous tissues.

The artificial neural network (ANN) is an artificial intelligence method that attempts to simulate the function of the human brain [6]. The convolutional neural network (CNN) is an artificial intelligence method that attempts to simulate the function of the human brain [6]. Based on the combination of biology and neurology, deep learning technology is a kind of the deep network model with hierarchical structure constructed by simulating the hierarchical working mode of the human brain visual system, which is inspired by the field of the human brain visual nerve [7]. What is more, the CNN is a derived ANN with the characteristics of hierarchical structure, extracting features, perceiving local areas, and classification due to a perfect combination of the ANN and deep learning technology [8]. The task requirement of modern image recognition is that the classification system can adapt to different kinds of recognition requirements, and the CNN has become a hot topic in the field of the ANN because of its high-efficiency recognition advantages. MRI is a medical imaging technique applied in radiology, which employs the combined action of a strong magnetic field, magnetic field gradients, and silent electric waves to form images of human organs to analyze the physiological processes or anatomy of the body image [9]. The radiomics is the most widely applied in the oncology, which includes tumor classification, shunt staging, and prognosis prediction. Ge et al. [10] combined the parameters of CT radiomics with clinicopathological characteristics for investigation, established a preoperative prediction model for EC, and verified the application value of this model in clinical diagnosis.

In this study, radiomics based on CNN modeling was adopted to intelligently identify the normal, hyperplastic, and cancerous tissues of the endometrium, providing a new method for clinical prediction of the emerging and development of EC.

## 2. Materials and Methods

### 2.1. Research Objects

In this study, 158 patients with EC, who underwent staged surgery in hospital from October 17, 2018, to May 21, 2020, were selected as the research objects and divided into the training group and the test group (79 cases in each group), with an average age of 56.9 ± 17.5 years. The medical ethics committee of hospital had approved this experiment, and each patient and his or her family members had understood the situation of this experiment and signed the informed consent form.

The criteria for inclusion were defined to include patients who were diagnosed with EC after surgery, had no contraindications to MRI scanning, were younger than 70 years old, and had clear consciousness for normal examination.

The criteria for exclusion were defined to include patients who suffered from mental disorders, had other malignant tumors such as cervical cancer, had incomplete clinical data, withdrew from this experiment due to their own reasons, and had poor MRI image quality for difficult recognition of the lesion.

### 2.2. Research Methods for Intelligent Recognition of Endometrial Cancer

Each patient underwent sagittal T1- and T2-weighted images of pelvic enhanced MRI before surgery. The CNN model was constructed, the imaging model for EC prediction was screened out based on features, and the comprehensive prediction model for EC was established based on clinical pathological information and imaging parameters. The patient's region of interest (ROI) was drawn, and the AUC, sensitivity, specificity, and accuracy were applied to evaluate the diagnostic effect of the constructed model, and its effect was verified in patients of the test group.

### 2.3. Dynamic Enhancement Magnetic Resonance Scanning

In this study, the MR Prisma 3.0 magnetic resonance instrument produced by Siemens, Germany, was employed to examine the patients. Before the scanning, the examination procedure should be described in detail to the patients. They should be in the supine position and maintain steady breathing. After MRI scanning, a high-pressure syringe was adopted to inject a 0.2 mmol/L contrast enhancer gadolinium-diethylenetriamine pentaacetic acid (Gd-DTPA) through the back of the hand vein at an injection rate of 2.5 mL/s. Then, the same amount of normal saline was injected. The scanning parameters were as follows. The matrix was 251 × 251, the layer thickness was 3.5 mm, the field of view was 25 × 25 cm, the flip angle was 15°, and the layer spacing was 6.1 mm. The obtained dynamic enhanced magnetic resonance images were sent to the workstation, and the images were processed by Functool II software.

### 2.4. Steps of the Back-Propagation Algorithm

Under the principle of gradient descent, the back-propagation (BP) algorithm searched for the minimum value on the error surface. The iterative process of each BP was divided into two steps. The first step was that an output result was generated during propagation before inputting the data. The second step was that the corresponding weights in the network were adjusted by back propagation to compute errors. The feedforward process and BP process were alternated, and the error was less than the set value or the time of iterations that reaches a set value unless the output result of the network reached a preset condition. For the multicategory classification problem with *B* categories and *M* training examples, the error function is

(1) $$\begin{array}{c} F^{M}=\frac{1}{2}{\overset{M}{\underset{m=1}{\sum }}\overset{B}{\underset{k=1}{\sum }}\left(p_{k}^{m}-q_{k}^{m}\right)}^{2}. \end{array}$$

In equation (1), *p*_*k*_^*m*^ represents the target value corresponding to the *k*^th^ dimension in the *m*^th^ sample, and *q*_*k*_^*m*^ stood for the network output value corresponding to *k*^th^ dimension in the *m*^th^ input. The error of the whole dataset was the sum of all single data errors. The BP of a single sample could be expressed as the following equation.

(2) $$\begin{array}{c} F^{m}=\frac{1}{2}\overset{B}{\underset{k=1}{\sum }}{\left(p_{k}^{m}-q_{k}^{m}\right)}^{2}=\frac{1}{2}{\left\|p^{m}-q^{m}\right\|}_{2}^{2}. \end{array}$$

In equation (2), *p*_*k*_^*m*^ expresses the target value corresponding to the *k*^th^ dimension in the *m*^th^ sample, and *q*_*k*_^*m*^ stood for the network output value corresponding to *k*^th^ dimension in the *m*^th^ input. For a normal full connection layer, the partial derivative of *F* relative to corresponding network weight could be calculated by the following form of the back-propagation rule. The output equation of the input layer is as follows.

(3) $$\begin{array}{c} x^{r}=g\left(v^{r}\right),\text{there into }v^{r}=W^{r}x^{r-1}+c^{r}. \end{array}$$

In equation (3), *r* represents the current layer, the output layer was defined as the *R* layer, and the input layer was specified as the 1^st^ layer.

The basic idea of the gradient learning algorithm was to find the error, calculate the partial derivative of parameters in the CNN, and identify the “error” in the BP network as the error signal of each unit pair's deviation. Besides, the equation could be as follows.

(4) $$\begin{array}{c} \frac{\partial F}{\partial c}=\frac{\partial F}{\partial v}\frac{\partial v}{\partial c}=\delta . \end{array}$$

In equation (4), (∂*F*/∂*c*) represents the partial derivative of the error with respect to the network parameter, and (∂*v*/∂*c*) was equal to 1. Therefore, the error signal was equal to the error relative to all the input partial derivatives of a unit. For *R* layer of the input layer, the partial derivative equation is obtained as follows.

(5) $$\begin{array}{c} \delta^{R}=g^{\prime }\left(v^{R}\right)\circ \left(q^{m}-p^{m}\right). \end{array}$$

In equation (5), *R* represents the input layer, and “∘” expresses the point-by-point product. The partial derivative *δ*^*R*^ was back-propagated from the upper layer through the network, and its equation could be shown as follows.

(6) $$\begin{array}{c} \delta^{r}={\left(w^{r+1}\right)}^{T}\delta^{r+1}\circ g^{\prime }\left(v^{r}\right). \end{array}$$

In equation (6), *δ*^*r*^ represents the partial derivative, and “∘” expresses the point-by-point product. Finally, the rule of the weight of a certain neuron for updating was that the neuron was input and multiplied by its triangular array. It was represented by a vector, which was the outer product of the input vector and the error signal vector, as shown in the following equations.

(7) $$\begin{array}{c} \frac{\partial F}{\partial W^{r}}=x^{r-1}{\left(\partial^{r}\right)}^{T}, \end{array}$$

(8) $$\begin{array}{c} \Delta W^{r}=-\xi \frac{\partial F}{\partial W^{r}}. \end{array}$$

Corresponding to the deviation *c* of equation (4), each weight *W*_*ij*_ usually had a corresponding *ξ*_*ij*_ in practical applications.

### 2.5. Structure of the Convolutional Neural Network Model

The network structure of LeNet-5 was adopted in this study, and the input data were a matrix formed by 32 × 32 pixels. The first feature image layer included 6 feature maps, and a 5 × 5 window was applied to convolve the input image, so as to obtain a 28 × 28 feature map. Then, it entered the first downsampling layer, and the first feature image layer was for downsampling operations to obtain 6 feature maps with a size of 14 × 14. The C3 layer was a convolutional layer, and the size of its convolution kernel was 5 × 5, which was the same as that of the C1 layer. It entered the S4 layer to continue the downsampling operation. The S4 layer was for convolutional operation by the C5 layer, and a fully connected method was adopted to perform convolution operations on the convolution kernel of each C5 layer on the basis of the S4 feature map. The C5 layer included 120 feature maps with a size of 1 × 1, and finally, the process of feature extraction was ended. Then, the result of 1 × 10 result was eventually output through a fully connected network on the basis of the C5 layer. In the vector whose output was 1 × 10, the classification result output by the network was the position corresponding to the largest component (Figure 1).

### 2.6. Data Preprocessing and the Convolutional Neural Network Model

In order to accelerate the convergence speed of the training algorithm, data preprocessing techniques were often adopted, including noise removal, dimensionality reduction of input data, and deletion of irrelevant data. Balanced data were very crucial in classification, and it was often considered that the data in the training set should be approximately evenly distributed relative to the label category. In order to balance the dataset, some redundant classification data should be appropriately removed, and some classification data with rare examples should be supplemented as much as possible.

CNN applied the structure that was the same as that of LeNet-5, but the following modifications had to be made. First, the tanh function should be employed to the output values of all layers in the network in LeNet-5, including the output layer results in the interval [0, 1], and the activation function applied in the CNN was the sigmoid function. Second, the radial basis function network structure was adopted in LeNet-5, and the CNN output layer was connected with the C5 layer to omit the F6 layer, so as to employ the fully connected method. Third, LeNet-5 applied a special learning rate sequence, and the learning rate during CNN training was fixed at 0.002. Fourth, the input data size of LeNet-5 was 28 × 28, while the CNN adopted the border filling method to expand the size to 32 × 32.

### 2.7. Technical Process of Radiomics

There was the technical process of radiomics, including 4 steps. The first step was to acquire images. Up to now, the images applied in radiomics research included MRI, computed tomography (CT), positron emission tomography (PET), and ultrasound. The second step was the image segmentation. The ROI or focus was sketched to prepare for the next feature extraction. The frequently applied segmentation methods included automatic, manual, and semiautomatic segmentation. The third step was to extract the image features. The extraction of image features was one of the critical steps of radiomics, which was to extract image features from the segmented ROI with high throughput to achieve the transition from image to quantitative data. At present, image extraction features contained morphological features and nonmorphological features. Morphological features described the shape, size, and location of lesions through traditional imaging methods. In addition, nonmorphological features included first-order, second-order, and high-order features. First-order features described the statistical distribution of each voxel, such as statistical features (mean, median, and skewness) generated through histograms; second-order features were texture features that described the relationship between voxels and reflect tumor abnormalities; and high-order features included wavelet features and fractal analysis. The fourth step was to analyze data and build models. The extracted image features were combined with statistics, pathological features, clinical data, and other information to construct an imaging prediction model that was suitable for clinical application. The specific radiomics flowchart is shown in Figure 2.

### 2.8. Statistical Methods

The data processing of this study was analyzed by SPSS19.0 version statistical software. The measurement data conforming to the normal distribution were expressed by the mean ± standard deviation ($\bar{x}$ ± *s*), and the nonconforming measurement data were represented by frequency (%). The accuracy, sensitivity, and specificity were collected in the prediction of the radiomics model and the comprehensive prediction model. *P* < 0.05 revealed that the difference was statistically obvious.

## 3. Results

### 3.1. Feature Distribution of all Patients

The patients were grouped into the training group and the test group, so as to investigate the feature distribution of patients in the two groups. There was no statistical difference in the feature distribution among patients in the two groups.  Figure 3 shows the comparison results of high-risk and low-risk data of preoperative biopsy pathology among patients in both groups. Moreover, there were comparisons on the normal and rising levels of CA125 in serums among patients in the two groups (Figure 4).

### 3.2. Imaging Features of Endometrial Cancer

The MRI imaging manifestations of each stage of EC were best shown on sagittal T2WI, which could clearly reflect the anatomical structure of the uterus. The typical manifestations were as follows. The endometrium was widened, the endometrial cavity was expanded, there were medium or low signal areas mixed with nodules in the high signal endometrial cavity, and larger masses presented different signal intensities due to necrosis, bleeding, and other reasons.

Endometrial hyperplasia was manifested as diffuse lesions in the uterine cavity, the endometrial was uniform and extensively thickened, diffusion weighted imaging (DWI) showed slightly high signal, and the endometrial thickening was limited and asymmetric (Figure 5). Endometrial polyps appeared as nodules or masses in the uterine cavity, showing a woven mesh-like uneven high signal on T2WI, and DWI indicated a slightly high signal (Figure 6). The T2WI of submucosal fibroids was like circular low signal, or nodules or tumors were dominated by low signal, and the surrounding boundary was light. If uterine bleeding was caused in the early stage, the surrounding boundary of the tumor would be unclear (Figure 7).

### 3.3. Experimental Results of the Convolutional Neural Network in Dataset

The network structure of the CNN was similar to that of LeNet-5. The main difference was that the CNN did not adopt some of the previous parameters in LeNet-5 and applied a fully connected network in the final classifier part. The misclassification rate curve of the CNN in the training process is shown in Figure 8. The abscissa stood for the times of iterations, and the ordinate represented the misclassification rate. The test misclassification rate after the CNN convergence was higher than that of LeNet-5, and the CNN test misclassification rate and training misclassification rate were higher than those of LeNet-5 during the entire training process.

### 3.4. Predictive Efficacy of the Radiomics Model

The prediction efficacy of the radiomics model of patients in the two groups was compared, including the accuracy, sensitivity, and specificity of patients from the two groups in predicting EC before surgery. It was found that the accuracy and specificity of patients in the two groups were not large, and the difference was not statistically obvious (*p* > 0.05). In addition, the sensitivity of patients in the training group was sharply lower than that of the test group, and there was a statistically great difference (*p* < 0.05) (Figure 9).

### 3.5. Predictive Efficacy of the Comprehensive Predictive Model

There were comparisons on the prediction efficacy of the comprehensive prediction model of patients in both groups, including the accuracy, sensitivity, and specificity of patients in the test group and training group in predicting EC before surgery. As shown in Figure 10, the accuracy and specificity of patients in the two groups were not marked, with no statistically huge difference (*p* > 0.05), while the sensitivity of patients in the training group was dramatically higher than that of the test group, and the difference was statistically substantial (*p* < 0.05).

### 3.6. Comparison on the Area under the Working Characteristic Curve of the Radiomics Model and Comprehensive Prediction Model

The AUC of the radiomics model was 0.897 in the training group and that of the comprehensive prediction model was 0.913 in the training group. It indicated that the two models constructed in this study had good prediction performance, and the effect of the comprehensive prediction model was better than that of the radiomic model. The AUC of the radiomics model and comprehensive prediction model in the test group was 0.889 and 0.897 in turn, which was similar to the above results. Therefore, it revealed that both models had great predictive performance, which again verified that the effect of the comprehensive prediction model was superior to the radiomics model (Figures 11 and 12).

## 4. Discussion

The etiology of EC has not been clear up to now. Metin et al. [11] employed the radiomics to establish a preoperative predictive model of EC. The radiomics preoperative prediction research also had been reported in the early cervical cancer [12] and bladder cancer [13]; the radiomics models of these research were the images based on different sequences of CT or MRI. Moreover, some other clinical pathological information was integrated. They could achieve the ideal prediction, which was consistent with the results of this study. The comprehensive prediction model was constructed in this study by combining specific imaging parameters with clinical pathological information. The results showed that the prediction performance was great and confirmed in the test group, indicating that the imaging parameters could be used as noninvasive markers for the prediction of EC.

In the research of EC, Takagi et al. [14] evaluated EC through the prediction model based on PET. It was found that PET was not suitable for routine examination of EC. Xuet al. [15] analyzed the single texture features of EC based on the MRI model, without complete radiomics analysis and independent risk factor validation. In this study, EC was for the complete MRI radiomics analysis under the CNN-based BP algorithm. From the results, the established model could achieve good specificity and sensitivity, which was superior to the above two models.

In this study, the diagnostic efficacy of the comprehensive predictive model in the training group and the test group was higher than that of the radiomics model, indicating that the diagnosis of disease required the comprehensive evaluation of clinical pathological features, pathological information, and various data of the radiomics. On the basis of the development of the CNN and the famous LeNet-5, a simple neural network model was constructed and applied to the identification of EC. The experimental results revealed that the simplified structure of the CNN could also achieve a better classification identification rate.

## 5. Conclusion

The enhanced MRI imaging analysis was for preoperative pelvic cavity in patients with EC based on radiomics of the CNN, the CNN model of preoperative EC was constructed, and the imaging specific parameters were combined with the clinical pathological information to establish the comprehensive prediction model. The results indicated that the prediction performance of the above models was good and verified in the test group, suggesting that the model constructed in this study could be applied in clinical practice. The limitations of this study were that all subjects came from the same hospital, MRI images were all from the same instrument, and the number of samples was also limited. Furthermore, the production of cancer markers was not taken into account during the research, so further investigation was needed. To sum up, the CNN model constructed in this study could be adopted to the clinical prediction and diagnosis of EC by radiomics analysis.

## Figures and Tables

**Figure 1:** The structure of the CNN model.

**Figure 2:** Technical process of radiomics.

**Figure 3:** Pathological comparison of preoperative biopsy among patients in the test and training groups.

**Figure 4:** Comparison of CA125 levels in serums from patients.

**Figure 5:** The image of endometrial tissue hyperplasia.

**Figure 6:** The image of endometrial polyps.

**Figure 7:** The image of endometrial tissue submucosal fibroids.

**Figure 8:** Comparison of the CNN and LeNet-5 misclassification rate trend.

**Figure 9:** Comparison on prediction efficiency of the radiomics model. (Note:  ^*∗*^The difference was statistically substantial in contrast to the sensitivity of the training group (*p* < 0.05).).

**Figure 10:** Comparison on prediction efficiency of the comprehensive prediction model. (Note:  ^*∗*^A statistically great difference in contrast to the sensitivity of the training group (*p* < 0.05).).

**Figure 11:** The AUC of the radiomics prediction model in the two groups.

**Figure 12:** The AUC of the comprehensive prediction model in the two groups.

## Data Availability

The data used to support the findings of this study are available from the corresponding author upon request.
